The article "Preparation of Curcumin Solid Lipid Nanoparticles Loaded with Flower-Shaped Lactose for Lung Inhalation and Preliminary Evaluation of Cytotoxicity In Vitro" was retracted in 2023. Reasons: signs of a paper mill; compromised peer review; unreliable results or conclusions.

# Preparation of Curcumin Solid Lipid Nanoparticles Loaded with Flower-Shaped Lactose for Lung Inhalation and Preliminary Evaluation of Cytotoxicity In Vitro

**DOI:** 10.1155/2021/4828169

**Published:** 2021-10-28

**Authors:** Nan Li, Xu Li, Peng Cheng, Ping Yang, Pengcheng Shi, Lingyu Kong, Hongbin Liu

**Affiliations:** ^1^Pharmaceutical Analysis Center of Tianjin Institute of Medical and Pharmaceutical Sciences, 79 Duolun Road, Heping District, Tianjin 300020, China; ^2^Cardiovascular and Cerebrovascular Drugs Research and Development Center of Tianjin Institute of Medical and Pharmaceutical Sciences, 79 Duolun Road, Heping District, Tianjin 300020, China; ^3^Tianjin Institute of Medical and Pharmaceutical Sciences, 79 Duolun Road, Heping District, Tianjin 300020, China; ^4^Oncology Drug R&D Center of Tianjin Institute of Medical and Pharmaceutical Sciences, 79 Duolun Road, Heping District, Tianjin 300020, China

## Abstract

The purpose of this study is to design a flower-shaped lactose loaded curcumin solid lipid nanoparticles dry powder inhaler and characterize it to improve the solubility and dissolution rate of curcumin in lung. Curcumin solid lipid nanoparticles (Cur-SLNs) were prepared by solvent evaporation method, and then they were micronized by freeze-drying technology. Finally, Cur-SLN micropowder obtained by freeze-drying was mixed with flower-shaped lactose (FL) at a ratio of 2 : 1 and then passed through a 200-mesh sieve to obtain Cur-SLN-FL powder. Tween-80 was selected as the surfactant to inhibit the aggregation of drug solid lipid nanoparticles. Under the optimum conditions, the solid lipid nanoparticles (SLN) were relatively spherical, with an average particle size of 14.7 nm, narrow distribution, Zeta potential of −22.5 mV, encapsulation efficiency of 90.21%, and drug loading of 8.56%. According to the particle size, PI, Zeta potential, drug loading (LC%), encapsulation efficiency (EE%), morphology, and in vitro release characteristics, the prescription of solid lipid nanoparticles was screened. Dry powder inhaler (DPI) was characterized by differential scanning calorimetry, scanning electron microscopy, particle size, density, and in vitro release performance. Its cytotoxicity to mouse fibroblasts (L929) and human normal lung epithelial cells (BEAS-2B) in vitro was investigated, and its safety for pulmonary inhalation was preliminarily determined. FTIR analysis shows that the micronized Cur-SLN-FL has the same chemical structure as FL. FTIR and DSC analysis confirmed that the characteristic absorption peak of curcumin was not found in Cur-SLN-FL, showing similar structure to SLN and FL. In addition, curcumin was coated in solid lipid nanoparticles to make powder mist, which increased its drug loading, kept its aerodynamic particle size (4.03 ± 0.40) *μ*m, and significantly improved its drug release performance in artificial lung fluid. In vitro cytotoxicity test results confirmed that Cur-SLN-FL was less toxic to BEAS-2B cells than L929 cells. Therefore, curcumin was prepared into solid lipid nanoparticles by emulsion evaporation-low temperature solidification method and then micronized and mixed with FL to prepare curcumin solid lipid nanoparticle powder mist loaded with flower-shaped lactose. The process is simple and feasible, and it has better safety performance for lung cells, which is expected to become a safe and effective delivery system for pulmonary inhalation drugs.

## 1. Introduction

In recent years, with the aggravation of environmental pollution, especially air pollution (PM_2.5_ particles), high smoking rate, and aging population, respiratory diseases caused by this are consuming more and more lives. Chronic obstructive pulmonary disease (COPD) is an inflammatory disease characterized by incomplete reversible airflow restriction [1]. Chronic inflammation of the airway is the main feature of COPD. Recent studies have found that overactivation of Nod-like receptor protein NLRP3 Inflammasome body plays an important role in the development of chronic inflammation of COPD [2]. Curcumin (Cur) is an important active polyphenol extracted from *Curcuma*, which can play a significant role in the treatment of COPD through anti-inflammation [3, 4]. A recent study on the diet of the elderly in Asia confirmed that eating more curcumin can significantly improve lung function, thus reducing the risk of COPD [5]. Studies have shown that curcumin has a significant inhibitory effect on NLRP3 infection, such as alleviating kidney injury by inhibiting NLRP3 infection [6], inhibiting the activation of NLRP3 Inflammasome corpuscles in endothelial cells to prevent and treat cardiovascular diseases, and so forth [7]. However, whether curcumin has a therapeutic effect on COPD by inhibiting the activation of NLRP3 infection has not been reported.

Anti-inflammatory therapy is the basic treatment principle and method for COPD at present. Its treatment strategy is to improve the lung function and reduce inflammation. Intravenous administration is the main treatment in acute stage, and inhalation administration is the first choice in stable stage. Inhaled glucocorticoid combined with long-acting *β*_2_ receptor agonist can effectively reduce inflammation and improve lung function. However, the dose-effect relationship and long-term safety of inhaled glucocorticoids are still unclear, and the side effects such as increased risk of infection cannot be ignored [8].

Sustained-controlled release inhalation drug delivery system can control the local or systemic release of drugs, so as to achieve the effect of reducing drug delivery times and side effects [9]. Dry powder inhaler (DPI) is composed of drug molecules and carrier particles, and the carrier used as DPI has strict size requirements, which must be a material that can be absorbed by respiratory tract and lung cells or has no influence on them. Considering the size of airway in lung, the form of drug or carrier material should be 1∼5 *μ*m particles [10].

Because Cur has a short half-life, is insoluble in water, and is easy to hydrolyze in neutral and alkaline environments, how to improve the solubility, bioavailability, and stability of curcumin has become the key to solve the clinical application of curcumin [4]. In the previous research, curcumin solid lipid nanoparticles (Cur-SLNs) were prepared by microemulsion method. Cur-SLN-DPI was obtained by micronizing Cur-SLN and mixing it with carrier InhaLac® 230 and the third component [11, 12]. During the research, we found that lactose monohydrate will fix the drug molecules through molecular adsorption, so it has the universality of powder mist agent, and the separation efficiency of the drug from the carrier is low. The lactose in the dry powder composition cannot enter the bronchioles because of its particle size >5 *μ*m, so how to desorb the drug becomes one of the important factors to improve the deposition rate of the effective parts of the drug.

Flower-shaped lactose (FL) is made of pure lactose (the only DPI safety carrier authorized by FDA), which can be customized in size, and has flower-shaped appearance, high uniformity, and obvious porous structure inside. Compared with conventional inhaled lactose, the flower-shaped particles with nanopores have a large surface area, with an average size (SMD) of 4.88 *μ*m and an aerodynamic size of 2.31 *μ*m. XRD crystallization test shows that it is in *α*/*β* compound crystalline state. In air water absorption test, it is similar to lactose monohydrate (crystalline state) but different from amorphous lactose. In water solubility test, FL is extremely soluble in water (30 s dissolution test), and its water solubility rate is comparable to amorphous lactose [13].

Solid lipid nanoparticles (SLN) contain the advantages of liposome and nanoemulsion and have the characteristics of improving drug stability and hydrophilicity, prolonging half-life, releasing drugs locally, and improving bioavailability [14]. In this study, based on the optimization of SLN preparation process, a new Cur-SLN-FL loaded with FL was constructed, in order to achieve the targeting and long-term sustained-release effect of curcumin in lung. The cytotoxicity of Cur-SLN-FL in vitro was evaluated by mouse fibroblast (L929) cells and human normal lung epithelial cells (BEAS-2B), respectively, in order to provide a safe and efficient intrapulmonary drug delivery method for the treatment of COPD.

## 2. Instruments and Materials

### 2.1. Instruments

SPD-M20A ultraviolet detector is purchased from Shimadzu Company, Japan; LC-20A high performance liquid chromatograph and IRAffinity-1S infrared spectrometer were purchased from Shimadzu Company, Japan. The AB135 one-tenth electronic balance and AL204 one-tenth electronic analysis day are purchased from Mettler Toledo Company in Switzerland on average; FDU-2110 freeze dryer was purchased from EYELA company in Japan; SZ-100 nanoparticle size analyzer was purchased from Horiba Company, Japan. Type 214 differential scanning calorimeter was purchased from HETZSCH company in Germany; H-7650 transmission electron microscope was from Hitachi Ltd., Japan; S-3400N scanning electron microscope was purchased from Hitachi, Japan; HELOS-OASIS laser particle size analyzer was purchased from Sympatec Company in Germany; Sigma-3k30 high-speed freezing centrifuge was purchased from Sigma-Aldrich Company in Germany. Amicon Ultra-15 centrifugal ultrafiltration tube was from Millipore (100 kDa MWCO, Ireland); Sorvall Legend 17R microcentrifuge was purchased from Thermo Fisher Scientific Company, USA.

### 2.2. Main Drugs and Reagents

Curcumin bulk drug (batch number TZSW200317-1, purity 99.0%) was purchased from Xi'an Tongze Biotechnology Co., Ltd.; curcumin reference substance (batch number 110823-201004, purity 99.0%) was purchased from China Food and Drug Administration Research Institute. FL (batch number 20200312) was made in laboratory; stearic acid and absolute ethanol (batch numbers 20191102 and 20200726) were purchased from Tianjin Chemical Reagent Wholesale Company; Polysorbate 80 (batch number 20191209) was purchased from Tianjin Guangfu Fine Chemical Research Institute; fetal bovine serum was purchased from PAN company in Germany; streptomycin mixture and 0.25% trypsin were purchased from HyClone Company. MEM culture solution was purchased from CORNING Company. Methanol and acetonitrile are chromatographically pure, other reagents are analytically pure or commonly used in laboratory, and water is Wahaha purified water.

### 2.3. Cell Lines

L929 cell line (mouse fibroblast cell line) was purchased from the cell bank of the Chinese Academy of Sciences; BEAS-2B was purchased from American Type Culture Collection (ATCC).

## 3. Methods and Results

### 3.1. Determination Method of Curcumin in Cur-SLN

#### 3.1.1. Determination of Curcumin Content

The content of curcumin was determined by HPLC.

#### 3.1.2. Chromatographic Conditions

Chromatographic column is Agilent C_18_ column (150 mm × 4.6 *μ*m, 5 mm). The mobile phase was acetonitrile-glacial acetic acid (5%) aqueous solution (55 : 45, V/V). The detector is an ultraviolet detector; the detection wavelength is 426 nm; the flow rate is 1.0 mL/min; column temperature is 35°C; the injection volume is 20 *μ*l.

Because curcumin is unstable and easy to decompose when exposed to light, brown volumetric flasks are used during the experiment, and care should be taken to avoid light.

#### 3.1.3. Investigation of Linear Relationship

Accurately weigh the curcumin reference substance in a 50 mL brown volumetric flask, dissolve it with absolute ethanol, and make a standard stock solution containing curcumin of 127 *μ*g/ml. Then, accurately absorb different volumes of Cur standard stock solution into a 10 ml brown volumetric flask, and adjust the volume with absolute ethyl alcohol to prepare the solutions with the concentrations of 0.1277 *μ*g/ml, 0.6386 *μ*g/ml, 1.2771 *μ*g/ml, 6.3855 *μ*g/ml, 12.771 *μ*g/ml, 19.1565 *μ*g/ml, 31.9277 *μ*g/ml, and 63.855 *μ*g/ml. According to the chromatographic conditions in “3.1.2,” the standard curve was drawn with the mass concentration (*X*, mg/ml) of curcumin reference solution as the abscissa and the peak area (*Y*) as the ordinate, and the linear regression equation was *Y* = 108354*X* − 33943 (*r* = 0.9996), and the linear range of the detected mass concentration of curcumin was 0.1996. In precision test, RSD of curcumin peak area was 0.72% (*n* = 6). In the stability (24 h) test, RSD of curcumin peak area was 0.11% (*n* = 6). RSD of curcumin content in repeatability test was 1.31% (*n* = 6). Take 9 samples of Cur-SLN-FL test solution, and put them into 10 ml brown volumetric flask to prepare three samples with high, medium, and low concentrations, each with 3 samples. The average recoveries are 99.12%, 98.83%, and 99.31%, and the RSD is 0.43%, 0.78%, and 0.84% (*n* = 3).

### 3.2. Preparation of Curcumin Solid Lipid Nanoparticles by Solvent Evaporation Method

In this study, Cur-SLNs were prepared by solvent emulsification diffusion-low temperature curing method [15]. The specific methods are as follows: accurately weigh the prescribed amount of poloxamer 188 and tween-80, and add 72 ml pure water under constant temperature and magnetic stirring at 75°C and 540 r/min to completely dissolve it as water phase. In addition, the prescription amounts of curcumin, glyceryl monostearate, and PEG-40 stearate were accurately weighed, and 24 ml of absolute ethyl alcohol was added at the same temperature and rotation speed, and the organic phase was completely dissolved by magnetic stirring at constant temperature. At 80°C and 1020 r/min, the organic phase was slowly injected into the water phase under constant temperature magnetic stirring. After dropping, the organic phase was continuously stirred at constant temperature for 3 hours to concentrate it to 40 ml. Hot emulsion was added to cold water at 0∼2°C at a ratio of 1 : 1 (V/V) while it was hot and cured at low temperature for 2 h to obtain yellow Cur-SLN suspension, which was passed through a 0.45 *μ*m microporous membrane to obtain Cur-SLN suspension, and stored at 4°C for later use.

The method of blank SLN is the same as above except that no medicine is added, and the blank SLN suspension with light blue opalescence can be obtained.

### 3.3. Single Factor Investigation on Preparation of Cur-SLN

Preparation of SLN by solvent emulsification diffusion-low temperature solidification is a simple and controllable preparation method. Solid lipid material is dissolved in ethanol under heating condition and injected into heated dispersion medium containing a certain amount of surfactant to form colostrum under a certain magnetic stirring state. In the process of colostrum formation, the ethanol solution diffuses into the water phase, and the oil droplets formed under heating can be stabilized by the surfactant in the dispersion medium. The particle size of SLN prepared by this method is about 20 nm, with good dispersity and narrow particle size distribution.

On the basis of previous research and pretest, single factor investigation was carried out according to the preparation method under “3.2.” In the single factor investigation, 66 mg Cur, 400 mg glyceryl monostearate, 800 mg PEG-40 stearate, 24 ml absolute ethyl alcohol, the concentration of mixed surfactant in water phase (0.75%, m/v, in which the mass ratio of poloxamer 188 to tween-80 is 1 : 2), and 72 ml pure water were fixed.

#### 3.3.1. Influence of Temperature on SLN Quality

When preparing SLN, it is necessary to ensure that the solid lipid material at the preparation temperature is in a liquid state, so as to form small oil droplets under the action of mechanical stirring, and stabilize the newly formed small oil droplets under the action of surfactant, and then stand at room temperature, and the liquid lipid solidifies into solid lipid to form SLN. Therefore, the temperature of preparing SLN is an important parameter. In this experiment, we conducted a single factor investigation on the temperature of preparing SLN and evaluated the quality of SLN prepared at different temperatures with the particle size and distribution as the investigation index. The results are shown in Table 1.

It can be seen from the results in Table 1 that when the temperature is low (60°C), the size of SLN is larger and the size distribution is wider. With the increase of preparation temperature, the particle size of SLN decreases gradually and the particle size distribution narrows. When the temperature rises further (90°C), the particle size of SLN does not decrease obviously, but the distribution of particle size widens slightly. The analysis reason may be that when the temperature is low, the lipid material may solidify in the injection process, which leads to the lipid material not being in liquid form well in the preparation process, so the particle size of the prepared SLN is too large, which is not conducive to emulsification. When the temperature rises, the lipid material can be emulsified into liquid oil droplets, so the prepared SLN has smaller particle size and narrower particle size distribution. However, when the temperature is too high, the size distribution of SLN becomes wider instead of decreasing obviously. It may be that the system temperature is too high, and the kinetic energy of particles increases during the solidification of SLN, which leads to mutual aggregation and uneven particles. To sum up, 80°C was finally selected as the preparation temperature of Cur-SLN.

#### 3.3.2. Influence of Stirring Speed of Injecting Ethanol into Organic Phase on SLN Quality

In the process of preparing SLN by emulsion evaporation-low temperature solidification, the solid lipid material (organic phase) dissolved by absolute ethanol must be dispersed under the action of certain mechanical force, and the dispersed oil droplets are injected into the water phase to be stabilized by surfactant. Therefore, the stirring speed of ethanol injection into lipid material has an important influence on the quality of SLN. Since the boiling point of absolute ethyl alcohol is 78.3°C, in order to prevent the volatilization of absolute ethyl alcohol from affecting the preparation of organic phase, the preparation temperature of organic phase (75°C) and stirring time (5 min) were fixed in this experiment, and the quality of SLN prepared at different stirring speeds was evaluated with the particle size and distribution as the inspection index. The results are shown in Table 2.

It can be seen from the results in Table 2 that when the stirring speed is low (200 r/min), the particle size of the prepared SLN is larger. With the increase of stirring speed (400 r/min), the particle size of SLN decreases obviously and the particle size distribution narrows. When the stirring speed increases further, the particle size of SLN changes little, but the particle size distribution tends to be uniform. When the stirring speed is 500∼600 r/min, the size of SLN is similar, about 20 nm, and the size distribution is narrow. After comprehensive consideration, 540 r/min was finally selected as the stirring speed for injecting ethanol into organic phase.

#### 3.3.3. Influence of Organic Phase Mixing Time on SLN Quality

Like stirring speed, the time of magnetic stirring, that is, the time of mechanical force, has an important influence on the quality of SLN. The preparation temperature (75°C) and stirring speed (540 r/min) were fixed, and the influence of different stirring time on the quality of SLN was investigated with particle size and distribution as indicators. The results are shown in Table 3.

It can be seen from the results in Table 3 that when the stirring time is short (1 min or 3 min), the prepared SLN has larger particle size and wider particle size distribution. When the stirring time is further increased (5 min or 7 min), the particle size of SLN decreases obviously and the particle size distribution narrows. With the further increase of stirring time, the particle size of SLN does not decrease obviously but increases slightly and the particle size distribution widens. The reason may be that when the stirring time is short, the mechanical stirring force is not enough to fully disperse the liquid lipid into uniform oil droplets. With the increase of stirring time, the particle size of SLN decreases obviously, which shows that the stirring at this time is enough to disperse the liquid oil phase into uniform oil droplets. When the stirring time is too long, the collision probability between droplets will increase, which will lead to the collision between newly formed uniform droplets and widen the particle size distribution. Therefore, considering comprehensively, the stirring time is set to 5 min.

#### 3.3.4. The Influence of Lipid Material Mass Ratio on the Mass of Solid Lipid Nanoparticles

Generally speaking, the difficulty of nanocarrier as drug delivery system lies in its low drug loading. The reason is that the concentration of nanodrug delivery system in solution state should not be too large; otherwise the whole solution system will be unstable [16].

In this experiment, the mass ratio of lipid material (glyceryl monostearate and PEG-40 stearate) of the solid lipid nanoparticle dispersion was investigated. Nanoparticle dispersions with different solid lipid ratios were prepared with the best preparation process parameters, and the quality of solid lipid nanoparticles was evaluated by particle size and distribution. The results are shown in Table 4.

The results in Table 4 show that when the lipids of the two lipid materials are relatively large, the particle size of nanoparticles is larger than about 100 nm, and the particle size distribution is wide. When the lipid ratio decreases, the particle size of solid lipid nanoparticles decreases obviously and the particle size distribution narrows. The reason may be that when the ratio of solid to lipid is appropriate, the space distance between particles in the prepared SLN solution is large. Because of the comprehensive effects of Brownian motion and surface charge, the whole nanoparticle solution system is relatively stable. During the solidification of liquid SLN, particles are not easy to collide with each other. When the mass ratio of solid lipid material is not suitable, the number of nanoparticles per unit volume increases, which leads to the probability of collision and flocculation. Therefore, these nanoparticles are easy to collide with each other and become large particles in the curing process, which leads to the larger particle size of SLN. After comprehensive consideration, it is finally determined that the lipid ratio of the prepared solid lipid nanoparticles is 1 : 2, the prepared nanoparticles are about 18 nm, and the particle size distribution is narrow.

#### 3.3.5. Influence of the Concentration of Mixed Surfactant in Water Phase on the Quality of Solid Lipid Nanoparticles

When preparing solid lipid nanoparticles, certain amounts of poloxamer 188 and tween-80 were added to the water phase to emulsify and stabilize the oil droplets. The amount of emulsifier plays an important role in the stroke of emulsion. We investigated the dosage of mixed surfactants poloxamer 188 and tween-80 in the preparation process. The mass ratio of fixed poloxamer 188 to tween-80 was 1 : 2, and the water solution of mixed surfactant with different concentrations was used as water phase to investigate its influence on the quality of solid lipid nanoparticles. The results are shown in Table 5.

It can be seen from the results in Table 5 that when the concentration of mixed surfactant is low (0.1%∼0.5%), the particle size of solid lipid nanoparticles is larger and the particle size distribution is wider. When the concentration was further increased to 0.75%, the particle size and distribution of solid lipid nanoparticles decreased gradually, and then even if the concentration of poloxamer 188 was increased, the particle size and distribution did not change much.

#### 3.3.6. Effect of Stirring Speed of Water Phase on the Quality of Solid Lipid Nanoparticles

When the organic phase is injected into the water phase, it must be stirred continuously and at a high speed, so that the thermal emulsion system can be uniform and stable. When organic phase is injected into water phase, the influence of different stirring speed of water phase on the quality of solid lipid nanoparticles is investigated. The results are shown in Table 6.

It can be seen from the results in Table 6 that when the stirring speed is too slow, the organic phase and the water phase will be mixed unevenly, the particle size will be relatively large, and the distribution will be wide, so that a stable emulsion cannot be formed and the stability will be poor. When the stirring speed is too fast, the morphology of particles will be destroyed, and more foams will be produced, which will affect the emulsifying effect of surfactants.

#### 3.3.7. Effect of Stirring Time of Emulsion Evaporation in Aqueous Phase on the Quality of Solid Lipid Nanoparticles

The process of injecting organic phase into water phase is carried out at constant temperature and constant rotation speed, and it is necessary to choose appropriate stirring time, which is helpful to form emulsion with stable state and uniform size. After the organic phase is injected into the water phase, the emulsion drops form immediately, and then it takes a certain time to make them fully dispersed and stabilized. We investigated the influence of stirring time of injecting organic phase into water phase to form emulsion on the quality of solid lipid nanoparticles, and the results are shown in Table 7.

It can be seen from the results in Table 7 that when the stirring time is short, the SLN formed has larger particle size and wider distribution, and the system is unstable and easy to produce flocculation after being placed. With the increase of stirring time, the particle size decreases gradually and the distribution narrows. After that, the stirring time continued to be prolonged, and the particle size and distribution of SLN had no obvious change. However, considering that the stirring time at high temperature was too long, curcumin was easily degraded, so this study chose 3 h as the stirring time for emulsification and evaporation.

Through the preparation technology of solid lipid nanoparticles and the single factor experimental results of each component affecting the quality of solid lipid nanoparticles, it is finally determined that the mixed surfactant aqueous solution with a concentration of 0.75% is used as the water phase; the lipid ratio is 1 : 2; emulsification temperature is 80°C; the stirring speed of organic phase preparation is 540 r/min; the stirring time of organic phase preparation is 5 min. The water phase emulsification evaporation stirring time is 3 h, and the stirring speed is 1020 r/min.

### 3.4. Optimization and Screening of Cur-SLN Prescription

According to the results of preexperiment and single factor experiment, four main factors affecting the quality of Cur-SLN were screened out, namely, emulsification evaporation temperature (*A*, °C), drug-lipid ratio (*B*), mass ratio of mixed surfactant poloxamer 188 to tween-80 (*C*), and freeze-curing stirring temperature (*D*). Selecting three levels for each factor, taking the average particle size and encapsulation rate as evaluation indexes, and using Orthogonal Design Assistant II v3.1 software, L9 (3^4^) orthogonal test (Table 8) was designed to optimize the best preparation process of curcumin solid lipid nanoparticles. The weighted analysis method was used to comprehensively analyze the orthogonal test results. The average particle size (*y*_1_) and the encapsulation rate (*y*_2_) were integrated by the coefficients of 55% and 45%, respectively, and the comprehensive bisection (*y*) was 55 (1 − *y*_1_/103.9) + 45 × *y*_2_/81.5 [17].

It can be seen from the experimental design results in Table 8 and the variance analysis results in Table 9 that the primary and secondary order of the four factors affecting the average particle size and encapsulation rate of Cur-SLN is *C* > *B* > *A* > *D*, and the best prescription is *A*_3_*B*_2_*C*_3_*D*_1_; that is, the emulsification evaporation temperature is 80°C, the ratio of medicine to fat is 1 : 6, F68-T80 (1 : 2), and the freeze-curing stirring temperature is 2°C.

### 3.5. Physical and Chemical Properties of Solid Lipid Nanoparticles

Three batches of Cur-SLN were prepared by the best preparation technology, and their average particle size and distribution, particle morphology, entrapment efficiency, and drug loading were determined.

#### 3.5.1. Particles Diameter, Polydispersity Index, and Zeta Potential

The main factors affecting the physical stability of solid lipid nanoparticles are particle size and surface charge [18]. Particle size, polydispersity coefficient (PI), and Zeta potential of Cur-SLN were evaluated by dynamic light scattering (DLS) technique and the scattering angle was 90°.

All samples were undiluted and tested directly at room temperature.

Average particle size, PI (Figure 1(a)), and Zeta potential (Figure 1(b)) of solid lipid nanoparticles obtained by the best preparation process were analyzed by SZ-100 nanoparticle sizer (Horiba, Japan). Means and standard deviations (mean ± SD) were calculated from three determinations. The results show that the size distribution of solid lipid nanoparticles prepared by this method is relatively uniform, and the average particle sizes of the three batches of samples are 17.4 nm, 18.1 nm, and 17.9 nm, with an average of 17.8 ± 0.36 nm, and the particle size distribution is narrow (PI: 0.144). The Zeta potentials were −22.6 mV, −23.1 mV, and −21.8 mV, with an average value of −22.5 ± 0.66 mV. According to bilayer theory, the Zeta potential is closely related to the stability of nanoparticle system. Theoretically, the Zeta potential is within −20∼−35 mV, and nanoparticles are relatively stable. The average Zeta potential of Cur-SLN prepared by the best preparation process has negative charge, strong repulsion, and good stability.

#### 3.5.2. Morphology Analysis

The morphological analysis of SLNs and Cur-SLNs was performed by transmission electron microscopy (TEM Hitachi H-7650; Hitachi Ltd., Japan). Take 20 *μ*l of the prepared solid lipid nanoparticle solution and drop it on the copper mesh, adsorb it for 5 min, and, after natural drying, cover the copper mesh on 2% phosphotungstic acid dyeing solution, dye it for 10 s, absorb phosphotungstic acid with filter paper, and then apply 80 kV accelerating voltage for analysis and image scanning. TEM is an effective analytical method to observe the morphology and structure of nanoparticles and the fine structure of biological samples. It can be seen from Figure 2 that the nanoparticles are spherical and elliptical solid particles.

#### 3.5.3. Encapsulation Efficiency and Loading Capacity

Encapsulation rate and drug loading are two important indexes to evaluate the preparation technology of a microparticle drug delivery system [11]. In order to determine the entrapment efficiency accurately, it is the key to separate nanoparticles from free drugs. Because nanoparticles are much larger than uncoated drug particles, they can be separated by their different sizes [19].

The entrapment efficiency of Cur-SLN was determined by ultrafiltration centrifugation; that is, 1 ml of Cur-SLN suspension was accurately weighed, put into a 25 ml brown volumetric flask, added with methanol for demulsification and dissolution, diluted to scale, shaken evenly, and extracted by ultrasonic for 15 min. Let stand, take the supernatant, and filter it through a 0.45 *μ*m microporous membrane, take the filtrate for determination, measure the Cur peak area by HPLC, and calculate the Cur content in the sample. In addition, Cur-SLN samples with the same volume were accurately measured in the upper part of ultrafiltration centrifuge tube and centrifuged for 10 min at 4°C and 14000 r/min. The nanoparticles were trapped on the filter membrane, and the free drug entered the filtrate. The nanoparticles and filtrate were extracted with methanol, diluted by a proper multiple, and passed through a 0.45 *μ*m microporous filter membrane to determine the content. See “3.1.2” for HPLC determination.

A standard curve was used to determine the concentration of curcumin and results are expressed as mean ± standard deviation (*n* = 3).

(1) $$\begin{array}{c} \text{EE }\%=\frac{\text{initial amount of cur}-\text{total free cur}}{\text{initial amount of cur}}\times 100,\\ \text{LC }\%=\frac{\text{amount of encapsulated cur}}{\text{total amount of lipid and drug}}\times 100. \end{array}$$

The encapsulation efficiency (EE%) and drug loading (DL%) of three batches of Cur-SLN-FL were 90.21 ± 1.12 (%) and 8.56 ± 0.87 (%), respectively.

### 3.6. Study on Stability of Solid Lipid Nanoparticles

The stability of nanopreparation is the premise of developing a new drug delivery system. Because nanodrug delivery system is a particle dispersion system, that is, a thermodynamically unstable system, the stability of SLN suspension in liquid state is worse than that of solid preparation [20]. The physical stability of Cur-SLN stored at room temperature (25°C) and low temperature (4°C) was investigated with the average particle size and Zeta potential as indexes, and the results are shown in Figure 3.

As shown in Figure 3(a), under the storage condition of low temperature (4°C), the particle size of SLN did not change obviously within 14 days but increased slightly with the extension of time (28 days). However, at room temperature (25°C), the particle size of SLN did not change significantly within 7 days but increased significantly with the extension of time (7–28 days), with slight flocs at the bottom, which could be redispersed after shaking. The above experimental results show that the solid lipid nanoparticles are relatively stable in the solution system, and the stability at low temperature (4°C) is better than that at room temperature (25°C). The size of SLN prepared in solution state (4°C) can be kept unchanged for 28 days.

Solid lipid nanoparticles are mainly prepared from solid lipid materials. During storage, free fatty acids may be produced due to oxidation or biodegradation, which may lead to changes in the surface potential of nanoparticles. The potential change of SLN directly affects its physical stability, because nanoparticles can maintain the stability of the system only by maintaining a certain surface potential, and too large or too small surface potential is not conducive to the stability of the whole system. In this experiment, the Zeta potential of solid lipid nanoparticles under two different storage conditions was measured (Figure 3(b)). No obvious change in Zeta potential of solid lipid nanoparticles was observed within two weeks, whether at low temperature (4°C) or room temperature (25°C), which indicated that the whole system did not produce excessive free fatty acids during storage.

### 3.7. Freeze-Drying

Trehalose was used as freeze-drying protective agent (3%, w/v) for blank SLN and Cur-SLN to protect SLN from the mechanical stress of ice crystals.

The blank and drug-loaded nanosuspensions were, respectively, packed in glass watch glasses and put into the program freeze-drying chamber of freeze dryer (FDU-2110, EYELA, Tokyo, Japan) for program freeze-drying. The freeze-drying program was set as follows: S1: prefreezing at −35°C for 3 hours; S2: keep at −35°C and 2.1 Pa pressure for 9 h; S3: keep at −20°C and 2.1 Pa pressure for 12 h; S4: keep at −10°C and 2.1 Pa for 8 h; S5: holding at 0°C and 2.1 Pa for 8 h; S6: holding at 20°C and 2.1 Pa for 5 h; complete the drying of the sample. The freeze-dried powder obtained is light yellow, full in appearance, smooth surfaces, without shrinkage or collapse, uniform in color, and good in redispersibility. The average particle size of Cur-SLN powder after redissolving is 21.47 ± 1.14 nm, and the Zeta potential is −22.57 ± 0.46 mV, which indicates that the freeze-drying process does not destroy the structure and stability of Cur-SLN.

After freeze-drying, store all samples in a desiccator and keep them away from light.

### 3.8. Preparation and Characterization of Flower-Shaped Lactose Loaded Solid Lipid Nanoparticles

#### 3.8.1. Preparation of Flower-Shaped Lactose Loaded Solid Lipid Nanoparticle Dry Powder

Cur-SLN micro powder obtained after freeze-drying was mixed with FL at a ratio of 2 : 1 and then passed through a 200-mesh sieve to obtain Cur-SLN-FL powder mist agent.

#### 3.8.2. Fourier Transform Infrared Spectroscopy

The surface chemical properties of SLN-FL were studied by Fourier transform infrared spectrometer (FTIR). Use FTIR equipped with FTIR (IRAffinity-1S FTIR, Shimadzu, Japan) to evaluate Cur, SLN, Cur-SLN, and Cur-SLN-FL, weigh 2 mg of each sample and 300 mg of potassium bromide, respectively, and grind them evenly together. The ground sample was dried in an infrared dryer and then pressed under 20 MPa for 5 min to obtain the sample to be tested. Each sample to be measured is scanned in the wave number range of 4000∼500 cm^−1^ to obtain the corresponding spectrogram, and the infrared absorption peaks of each sample are compared and analyzed, respectively. The results are shown in Figure 4.

As shown in Figure 4, the infrared spectrum of Cur obtained in this study accords with the infrared spectrum of Cur recorded in the infrared spectrum library of the system, and there is an obvious characteristic peak at 1508 cm^−1^ [21]; FL particles have characteristic peaks at 3362 cm^−1^ and 1038 cm^−1^. Cur-SLN-FL and drug-free SLN-FL mainly show characteristic peaks similar to FL particles; that is, they have characteristic absorption peaks at 3364 cm^−1^ and 1037 cm^−1^ and 3361 cm^−1^ and 1038 cm^−1^, respectively, and there is no characteristic absorption peak of Cur. That Cur has been wrapped in SLN. On the other hand, Cur-SLN-FL and blank SLN-FL have similar characteristic peaks near 2900 cm^−1^ and 2386 cm^−1^, which may be the absorption peaks of SLN framework. Both of them show similar absorption characteristic peaks, which proves once again that the presence or absence of drugs has little effect on the surface chemical results of SLN-FL, and Cur has been encapsulated in SLN.

#### 3.8.3. Differential Scanning Calorimetry (DSC)

Use DSC 214 NETZSCH (NETZSCH, Germany) to perform differential scanning calorimetry (DSC) to determine the thermal transition properties of samples. 3 mg of Cur, SLN, Cur-SLN, and Cur-SLN-FL powders was put into a standard aluminum crucible, sealed, and punched. Take another empty crucible, cover it, seal it, and punch it as a reference. Differential scanning was carried out according to the test conditions (nitrogen purge flow rate is 60 mL/min, heating rate is 20°C/min, and heating range is −20∼350°C), and the results are shown in Figure 5.

According to the analysis of Figure 5, Cur has a characteristic absorption peak at 183.0°C, and two peaks appear at 101.3°C and 261.9°C. The FL particles have characteristic absorption peaks at 217.7, 231.1, 246.9, 302.0, and 335.8°C. However, the curves of SLN-FL and Cur-SLN-FL without drug loading are similar, and there is no characteristic absorption peak of curcumin. The characteristic absorption peaks of SLN-FL without drug loading are at 49.4, 93.7, 175.4, 217.2, and 252.4°C, and the two characteristic absorption peaks at 217.2 and 252.4°C are similar to FL. The characteristic absorption peaks of Cur-SLN-FL appear at 46.7, 100.6, 172.1, 277.3, 305.9, and 328.0°C, among which 46.7°C, 100.6°C, and 172.1°C are similar to SLN-FL, which may be the characteristic absorption peaks of SLN skeleton, while 305.9°C is similar to the characteristic absorption peak of FL particles. The above results suggest that Cur is encapsulated in SLN to make freeze-dried powder and then mixed with FL to form a new phase.

#### 3.8.4. Scanning Electron Microscopy (SEM)

The morphology of Cur-SLN-FL was observed and photographed by Hitachi S3400N (Hitachi, Tokyo, Japan). Coat SLN-FL (blank SLN) and Cur-SLN-FL on the metal plate which is fixed with double-sided conductive adhesive. Samples which can be observed by scanning electron microscope were prepared by spraying gold with electron beam for 40 mA and 20 min, and micrographs were taken under 5.0 kV voltage and different magnification to observe the morphology of the samples to be measured.

The results showed that SLN-FL (a) and Cur-SLN-FL (b) powder mist showed flower-shaped appearance (Figure 6). When the flower-shaped lactose is used as a carrier of the dry powder inhalant and mixed with the medicinal lyophilized powder, the flower-shaped lactose is adsorbed on the surface of the dry powder inhalant, so that the surface morphology of the Cur-SLN lyophilized powder is modified, and the roughness is increased.

#### 3.8.5. Particle Size

Particle size analysis was carried out with new Pataik HELOS-OASIS (SYMPATEC GmbH, Germany) dry disperser, and the test was repeated three determinations. Take a proper amount of Cur-SLN-FL powder, sieve it with 200-mesh sieves, run at 50% vibration rate and 2.0 bar dispersed air pressure, and measure the particle size of the powder. *X*_50_ is the median diameter representing the geometric diameter of particles.

Results show that Cur-SLN-FL has an average particle size (SMD) of 4.95 ± 0.57 *μ*m and a median geometric particle size (*D*_*e*_) of 7.66 ± 0.76 *μ*m, and the optimal particle size for macrophage endocytosis is 1∼3 *μ*m [22], so we prepared it for evaluation of particle size of powder mist agent by calculating aerodynamic particle size (*D*_*a*_); *D*_*a*_ is calculated according to the following formula:

(2) $$\begin{array}{c} D_{a}=D_{e}\sqrt{\frac{\rho_{p}}{\rho_{0}\chi }}. \end{array}$$

In the formula, *D*_*e*_ is the median geometric particle size; *ρ*_*p*_ is the effective particle density, and its value is 1.26 times that of tap density; *ρ*_0_ is the reference density, which is 1 g/cm^3^; *χ* is a dynamic morphological factor (*χ* = 1 when spherical, 1 is used in this paper). It is generally believed that aerodynamic particles with a particle size of 1∼5 *μ*m can reach deep lung [22, 23].

After calculation, *D*_*a*_ of Cur-SLN-FL powder aerosol prepared in this study is 4.03 ± 0.40 *μ*m, which is in the range of 1∼5 *μ*m, and is suitable for lung inhalation [24].

#### 3.8.6. Powder Properties of CUR-SLN-FL

*(1) Bulk Density*. According to the literature method, take a dry measuring cylinder (5 mL) and accurately weigh its mass (*m*_1_). Then accurately weigh an appropriate amount (about 1 g) of Cur-SLN-FL powder after passing through a 200-mesh sieve, accurately weigh its mass (*m*_2_), and read the powder volume (*V*) in the measuring cylinder. Calculate the bulk density of Cur-SLN-FL according to the following formula: bulk density = (*m*_2_ − *m*_1_)/*V*. Means and standard deviations (mean ± SD) were calculated from three determinations. The results showed that the bulk density of Cur-SLN-FL composite dry powder was 0.16 ± 0.01 g/cm^3^ (Table 10), which indicated that the powder structure was loose, which was beneficial to the atomization and dispersion of lung inhalation.

*(2) Tapping Density*. According to the literature method. Accurately weigh an appropriate amount of Cur-SLN-FL (about 1 g) after passing through a 200-mesh sieve, slowly add it into a drying measuring cylinder (5 ml), tap the powder in the measuring cylinder for 500 times, record the mass (*m*_1_) of the tapped powder, and read the powder volume (*V*) in the measuring cylinder. The tap density of Cur-SLN-FL powder is calculated according to the following formula: tap density = *m*_1_/*V*. The experiment was repeated three determinations. The results show that the tap density of Cur-SLN-FL powder is 0.22 ± 0.01 g/cm^3^ [25] (Table 10).

*(3) Angle of Repose*. The fluidity is directly related to the accuracy of dosing. Fixed funnel method was used for determination. Three funnels are connected in series and fixed at a height (*H*) about 1 cm away from horizontally placed paper. The sample powder is poured into the uppermost funnel along the funnel wall until the tip of the particle cone formed on the paper contacts the funnel mouth. The diameter (2*R*) of the cone bottom is measured and the angle of repose (*H*/*R*) is calculated. The experiment was repeated three determinations. The results show that the angle of repose of Cur-SLN-FL composite dry powder is 28.31 ± 0.42 (°) (Table 10), which indicates that it has good fluidity and is beneficial to ensure the accuracy of filling dose. The fluidity of Cur-SLN-FL dry powder prepared by us was preliminarily classified by measuring the angle of repose [12].

### 3.9. Moisture Determination

According to the second drying method of “0832 Moisture Determination Method,” the general rule of Chinese Pharmacopoeia (2015 edition), the moisture in samples was determined. Take 2 g of this product powder, spread it flat in a flat weighing bottle (thickness less than 10 mm) dried to constant quality, and weigh its mass (*m*_1_). Open the bottle cap, dry at 100∼105°C for 5 h, cover the bottle cap, transfer it to the dryer, let it cool for 30 min, and weigh its quality, Then dry at the above temperature for 1 h, let it cool, weigh the mass, and repeat the above drying and cooling operations until the difference between the weights weighed twice in succession does not exceed 5 mg, and the constant mass is taken as *m*_2_. According to the lost mass, calculate the water content of the sample: water content (%) = (*m*_1_ − m_2_)/*m*_2_ × 100%. The experiment was repeated 3 times. The results showed that the water content of Cur-SLN-FL powder was 6.37 ± 0.41 (%), which met the DPI stability requirement (the water content should not exceed 9.0%) [26].

### 3.10. In Vitro Drug Release Study

The release curve of Cur-SLN-FL was studied by simulating the drug release in lung environment. Artificial lung fluid (SLF) was prepared to simulate physiological conditions (lung environment with mucus).

#### 3.10.1. In Vitro Release Test

The SLF was prepared by referring to the literature [27].

Accurately weigh 1 mg of curcumin API and Cur-SLN-FL (including 1 mg of curcumin API), put them into 100 ml conical flask, add release medium (50 ml of newly prepared artificial lung fluid (SLF), respectively), and put the conical flask into a constant temperature oscillator with a rotating speed of 80 r/min and a temperature of 37°C. At 0.033, 0.083, 0.167, 0.25, 0.5, 0.75, 1, 1.5, 2, 4, 6, 9, 12, 18, 24, 36, and 48 h, 0.25 ml of artificial lung fluid was taken and supplemented with the same volume and temperature. The released liquid was centrifuged at 12000 r/min for 5 min, and the supernatant was absorbed. The mass concentration (*c*_*t*_) of curcumin in the solution at the corresponding time point (*t*) was determined by HPLC under “3.1.2,” and the cumulative release amount and cumulative release rate at each time point were calculated: cumulative release rate (%) = *M*_*t*_*/M*_0_, where *M*_0_ is curcumin content.

The dissolution curves of curcumin and Cur-SLN-FL powder in artificial lung fluid are shown in Figure 7. In SLF, Cur-SLN-FL has obvious sustained release effect compared with curcumin. There is an obvious sudden release phenomenon of API, which is close to 40% within 1 h, and reaches the plateau in about 6 h, with a cumulative release rate of 52.5%. Because curcumin is not stable to light and heat, yellow in the release solution obviously fades after 6 h, which suggests that curcumin may be degraded, and the cumulative release rate will not increase with time. Cur-SLN-FL powder released quickly in the early stage, with a cumulative release rate of 2.9% in 5 min, and then showed good slow release performance, until the cumulative release rate reached 86.2% in 72 h, which was about 1.64 times of curcumin. The results of artificial lung fluid release test showed that Cur-SLN-FL had the best release performance in artificial lung fluid. It is suggested that DPI prepared from API for pulmonary inhalation is more suitable for dissolution, absorption, and drug effect of curcumin in vivo, which may be related to the preparation process of artificial lung fluid simulating the physiological environment of human lung lining fluid and adding tween-80 to promote the dissolution of curcumin. At the same time, wrapping curcumin in SLN can protect API, with little influence of heat, pH, and photosensitivity.

#### 3.10.2. Fitting of In Vitro Release Model

The cumulative drug release curve of Cur-SLN-FL in artificial lung fluid was fitted by 0-order kinetic model, 1-order kinetic model, Higuchi model, Weibull model, and Ritger-Peppas model, and the results of drug release mechanism are determined in Table 11.

It can be seen from Table 11 that Weibull equation fits well in the in vitro release of curcumin in artificial lung fluid, with regression coefficient *R*^2^ of 0.9834, while Weibull model of Cur-SLN-FL has the highest fitting degree, *R*^2^ = 0.9962. It can be seen that the in vitro release process of Cur-SLN-FL accords with Weibull model, and there is a sudden release phenomenon of curcumin in artificial lung fluid at the initial release stage.

### 3.11. In Vitro Cytotoxicity Test

#### 3.11.1. L929 Cell Culture

Take out the cryopreservation tube from the liquid nitrogen tank, quickly put it into warm water, and shake it quickly until the cryopreservation solution is completely dissolved. Centrifuge at 1000 r/min for 5 min. The frozen solution was discarded, and the added cell culture solution was gently blown with a pipette to disperse the cells. Transfer the cell suspension to a culture bottle, add additional culture solution, loosen the bottle mouth, and culture in MEM culture solution containing 10% fetal bovine serum, 100 U/ml penicillin, and 100 *μ*g/ml streptomycin at 37°C in an incubator with 5% CO_2_ volume fraction.

#### 3.11.2. BEAS-2B Cell Culture

BEAS-2B cells were cultured in DMEM with 10% fetal bovine serum at 5% CO_2_ at 37°C, and the morphology and growth of cells were observed regularly under microscope CO_2_.

#### 3.11.3. Inoculation of Cells

L929 cells and BEAS-2B cells were cultured in DMEM containing 10% FBS and in 1640 medium containing 20% FBS, cultured in a cell incubator at 37°C and 5% CO_2_. When the cells grow to 70%–80%, they can be digested and passaged with 0.25% trypsin-EDTA solution.

#### 3.11.4. Detection of Cytotoxicity by LDH Method

On the day of inoculation, 1640 culture medium containing 10% FBS (L929 cells) and MEM culture medium containing 20% FBS (BEAS-2B cells) were used to prepare cell suspensions. The cell suspension with a density of about 5.0 × 10^4^ cells/mL was added to a 96-well culture plate, and 100 *μ*l was added to each well, which was cultured in an incubator for (24 ± 1) h.

100 *μ*l of Cur-SLN-FL extracts with different concentrations was added for treatment, and appropriate controls were set. After drug stimulation, the cell culture plate was centrifuged for 5 min with a perforated plate centrifuge, 400 g. Absorb the supernatant as much as possible, add 150 *μ*l of LDH release reagent provided by the kit diluted 10 times with PBS (add 1 volume of LDH release reagent to 10 volumes of PBS and mix well), shake the culture plate properly and mix well, and then continue to incubate in the cell incubator for 1 hour. Then, the cell culture plate was centrifuged with a perforated plate centrifuge, 400*g*, for 5 min. 120 *μ*l of supernatant from each well was added to the corresponding well of a new 96-well plate, and the absorbance was measured at 492 nm by microplate reader. Calculate cytotoxicity or mortality (%) according to the following formula:

(3) $$\begin{array}{c} Cytotoxicity=\frac{\text{absorbance of treated sample}-\text{absorbance of sample control hole}}{\text{absorbance of maximum enzyme activity of cells}-\text{absorbance of sample control hole}}\times 100. \end{array}$$

The results showed that IC_50_ values of Cur-SLN-FL in L929 cells and BEAS-2B cells were 2.20 mg/mL and 5.81 mg/mL, respectively.

## 4. Discussion

In our previous research, solid lipid nanoparticles were prepared by microemulsion method. The average particle size of SLN was 156.9 ± 2.2 nm, the polydispersity coefficient was 0.480, the Zeta potential was −24.8 mV, and the entrapment efficiency and drug loading of Cur-SLN were 87.73% and 7.72%, respectively. However, in the follow-up study, we found that it was easy to demulsify, the SLN formed was unstable, and the particle size distribution was uneven. In addition, higher concentrations of surfactants and cosurfactants are needed in the preparation process, so the entrapment efficiency and drug loading have little room for further increase. Therefore, in this study, the preparation process of SLN was investigated by emulsion evaporation-low temperature curing method. The use of mixed surfactants significantly improved the encapsulation efficiency, effectively reduced the particle size, reduced the aggregation of SLN, and greatly increased the stability and in vitro release of drugs [28].

It should be noted that when the hot emulsion is solidified at low temperature, it must be cooled quickly; otherwise, it may cause SLN to be easy to adhere and increase in particle size and be easy to settle, and the stability is not good. The stirring speed when the organic phase is injected into the water phase for dispersion and when the thermal emulsion is solidified and dispersed at low temperature is also an important factor affecting the particle size. When it is too slow, the particle size tends to increase, and its stability is poor. If it is too fast, more foams will be produced, which will affect the emulsifying effect of surfactants.

The release characteristics of Cur-SLN-FL are rapid release at the beginning and slow release at the later stage. Because of the large specific surface area of SLN and FL, a small amount of drug molecules will be adsorbed on the surface of SLN or enriched in the outer layer of SLN, and the free drugs in the outer layer and without encapsulation will be released quickly, resulting in the sudden release phenomenon in the initial stage of cumulative release curve.

After being deposited into the lung through respiratory tract, the drug particles first come into contact with the lung lining liquid, and the drug is dissolved and released from the deposited particles to participate in the absorption and transportation process in the lung. In this study, artificial lung fluid was used to simulate the contact process between Cur-SLN-FL deposited in respiratory tract and lung lining fluid. The surface body fluid of lung epithelium was about 20∼50 ml, with a large difference in thickness (0.07∼15 *μ*m) and a lung surface area of about 100 m^2^. Therefore, if the drug particles can be dissolved and released quickly after inhalation, the effective concentration of the drug in the focus area can be significantly increased. However, it should also be noted that the pulmonary environment is not completely the same as the simulated release environment in vitro, so the measurement results of in vitro release cannot completely reflect the release of Cur-SLN-FL inhaled and deposited into the lung, which needs to be confirmed by further study on the absorption and tissue distribution of Cur-SLN-FL inhaled into the lung.

In the early stage of this experiment, reducing disaccharides (sucrose and trehalose) were investigated as protectants, which can act as cryoprotectants in freezing process and dehydration protectants in drying and dehydration process. The addition of freeze-drying protectant can effectively prevent the direct contact between SLN during freeze-drying, which is not easy to break, and the oxidation and hydrolysis speed of drugs and lipids decreases. The outer surfactant and freeze-drying protectant molecules have hydrogen bond association, which plays the role of “pseudohydration layer,” forming low eutectic or glassy substance with water, inhibiting the growth of crystals, making ice crystals exist in microcrystalline or amorphous form, reducing their extrusion and mechanical damage to SLN, and effectively preventing freeze-drying process [29]. Compared with sucrose, trehalose has a higher glass transition temperature (120°C), so trehalose solution is less likely to form ice crystals. Moreover, trehalose also has magical hydration ability, and its solution can form a trehalose/water structure with stronger rigidity and stronger freeze dehydration resistance. The shape and performance of freeze-dried samples obtained in dry season are similar. However, in the wet season, sucrose is easier to absorb moisture, so the surface of samples obtained is not as uniform as trehalose as freeze-dried protective agent, and it collapses slightly after being placed at room temperature, which is not conducive to the preservation of freeze-drying [30]. Therefore, trehalose was selected as freeze-dried protective agent of SLN in this study.

There are many factors that affect the fluidity of powder, including particle type, average particle size, particle size distribution, moisture content, particle shape, specific surface area, density, storage time, and interaction between particles. Generally speaking, when the moisture content of powder is very low, the moisture is adsorbed on its surface, which has little effect on the fluidity of powder. With the increase of moisture, thin film water is formed around the adsorbed water; at this time, the relative movement between particles is not easy to occur, which limits the whole flow of particles. When the moisture increases beyond the maximum molecular bound water, the fluidity of powder becomes worse and even loses its fluidity. Therefore, the moisture content of the powder aerosol should be fully considered in the moisture-proof storage of the sample.

The application of engineered nanomaterials in medical treatment and diagnosis has led to the special dynamic behavior of nanoparticles including cellular uptake, transfer, and distribution to the nervous system and circulatory system, which has become a potential cause of their biological toxicity [31]. The lung is the target organ. When inhaled, small-sized nanoparticles can reach all parts of the respiratory tract through a diffusion mechanism, including the alveolar cavity [32]. Nanoparticles are deposited in the lungs; even if they are nontoxic or low-toxic fine particles, their ultrafine particles can also cause lung damage. At the same time, nanoparticles can enter the blood circulation through various ways. Particles retained in the airways or alveolar cavity may be swallowed by pulmonary macrophages or escape their surveillance, be absorbed by epithelial cells or enter the interstitium, and can pass through epithelial cells and vascular endothelial cells into blood circulation and lymphatic circulation and then be distributed to the whole body [31, 33].

Not only is the toxicity of nanoparticles limited to the dose-effect relationship but also nano-specific-effect relationships such as specific surface area and nanometer size may appear. The toxicity of nanoparticles is closely related to their own structural properties, including the size, surface area, charge, shape, and chemical composition of the nanoparticles, as well as the solution in contact with the nanoparticles, and the differences in cell animal models [34].

In this study, mouse fibroblast cells L929 and human normal lung epithelial cells BEAS-2B cultured in vitro were used as the research objects, and the toxic effect of Cur-SLN-FL prepared by us on cells was investigated. Safety and scientific and reasonable utilization provide theoretical basis. Lactate dehydrogenase (LDH) is widely present in biological cells. It is one of the enzymes contained in the cytoplasm of living cells. Under normal circumstances, it cannot penetrate the cell membrane. When cells are damaged, the permeability of the cell membrane changes, and LDH can leak into the extracellular medium and inhibit cell proliferation. We use the LDH method to make a preliminary assessment of cell viability.

## Figures and Tables

**Figure 1:** Measurement results of particle size and surface potential of solid lipid nanoparticles. (a) Particle size distribution diagram; (b) measurement results of surface charge.

**Figure 2:** A representative TEM image of Cur-SLN. Scale bar represents 100 nm.

**Figure 3:** Stability investigation of solid lipid nanoparticle suspension. (a) The particle size changes of solid lipid nanoparticles at low temperature (4°C) and room temperature (25°C) for different times; (b) Zeta potential changes of solid lipid nanoparticles at low temperature (4°C) and room temperature (25°C) for different time.

**Figure 4:** FTIR spectra of Cur, FL, blank SLN-FL, and Cur-SLN-FL.

**Figure 5:** DSC spectra: Cur, FL, SLN-FL, and Cur-SLN-FL.

**Figure 6:** A representative SEM image of Cur-SLN-FL. Scale bar represents 2.00 *μ*m.

**Figure 7:** Dissolution of curcumin and Cur-SLN-FL in simulated lung fluid.

**Table 1:** Effect of preparation temperature on particle size and distribution of SLN (*n* = 3).

Temperature (°C)	Size (nm)	PI (polydispersity index)
60	277.0	0.483
70	220.3	0.379
80	18.1	0.173
90	18.5	0.328

**Table 2:** Effect of stirring speed of injecting ethanol into organic phase on particle size and distribution of SLN.

Mixing speed (r/min)	Size (nm)	PI (polydispersity index)
180	333.7	0.315
300	218.7	0.327
420	141.6	0.333
540	19.1	0.187
660	17.3	0.172

**Table 3:** Effect of stirring time on particle size and distribution of SLN.

Stirring time (min)	Size (nm)	PI (polydispersity index)
1	317.8	0.373
3	195.0	0.316
5	18.8	0.159
7	64.8	0.270
10	90.5	0.294

**Table 4:** Effect of lipid ratio on particle size and distribution of solid lipid nanoparticles.

Lipid ratio	Size (nm)	PI (polydispersity index)
2 : 1	219.7	0.420
3 : 2	144.8	0.373
1 : 1	126.5	0.305
3 : 4	74.1	0.266
1 : 2	18.7	0.158

**Table 5:** Effect of dosage of poloxamer 188 on particle size and distribution of solid lipid nanoparticles.

Concentration of emulsifier (v/v) (%)	Size (nm)	PI (polydispersity index)
0.1	106.7	0.386
0.25	88.5	0.354
0.5	57.3	0.238
0.75	17.0	0.152
1.0	20.3	0.186

**Table 6:** Effect of stirring speed of water phase on particle size and distribution of solid lipid nanoparticles.

Speed of water phase (r/min)	Size (nm)	PI (polydispersity index)
840	88.5	0.336
1020	17.0	0.152
1200	20.3	0.186
1380	57.3	0.268

**Table 7:** Effect of stirring time of emulsification evaporation on particle size and distribution of solid lipid nanoparticles.

Time (h)	Size (nm)	PI (polydispersity index)
1	158.5	0.436
2	96.2	0.324
3	17.9	0.146
4	21.3	0.192

**Table 8:** The orthogonal design and result of the experiment.

No. of experiment	*A* (°C)	*B*	*C*	*D* (°C)	*y*_1_ (nm)	*y*_2_ (%)	*y*
1	70	1 : 3	2 : 1	2	154.2	69.3	11.63
2	70	1 : 6	1 : 1	10	79.3	73.1	53.38
3	70	1 : 9	1 : 2	25	62.5	78.2	65.09
4	80	1 : 3	1 : 1	25	58.3	80.7	68.70
5	80	1 : 6	1 : 2	2	18.1	89.2	94.67
6	80	1 : 9	2 : 1	10	123.6	76.5	31.81
7	90	1 : 3	1 : 2	10	56.2	79.1	68.93
8	90	1 : 6	2 : 1	25	78.9	82.3	58.68
9	90	1 : 9	1 : 1	2	106.7	62.4	32.97
*K*_1_	43.367	49.753	34.040	46.423			
*K*_2_	65.060	68.910	51.683	51.373			
*K*_3_	53.527	43.290	76.230	64.157			
*R*	21.693	25.620	42.190	17.734			

**Table 9:** Variance analysis data.

Source	Sum of square of deviations	Variance	*F* ratio	Significance
*A*	706.844	2	1.407	None
*B*	1065.137	2	2.120	None
*C*	2693.822	2	5.362	None
*D* (error)	502.39	2	1.000	None

*F*_0.05_ (2, 2) = 19.000.

**Table 10:** Characteristics of Cur-SLN-FL dry powder inhalation. *n* = 3, $\bar{x}\pm s$.

Group	Characteristics of dry powders					
	Bulk density (g·cm^−3^)	Tap density (g·cm^−3^)	Angle of repose (°)	SMD (*μ*m)	*D*_*e*_ (*μ*m)	*D*_*a*_ (*μ*m)
Cur-SLN-FL	0.16 ± 0.01	0.22 ± 0.01	28.31 ± 0.42	4.95 ± 0.57	7.66 ± 0.76	4.03 ± 0.40

**Table 11:** The regression of Cur and Cur-SLN-FL release in vitro.

Model	Formulations	Regression equation	*R* ^2^
Zero-order	Cur	*Q* = 35.2270 + 0.5526*t*	0.4646
	Cur-SLN-FL	*Q* = 15.1923 + 1.3381*t*	0.8471
First-order	Cur	Ln (1 − *Q*) = −48.6088 − 2.1597*t*	0.7046
	Cur-SLN-FL	Ln (1 − *Q*) = −85.3562 − 0.0600*t*Lnln [1/(1 − *Q*)] = 0.0421ln*t* + 81.7840	0.9770
Higuchi	Cur	*Q* = 4.5382*t*_1/2_ + 29.5309	0.7018
	Cur-SLN-FL	*Q* = 11.5534*t*_1/2_ + 0.6640	0.7204
Weibull	Cur	*Q* = 53.2737 (1 − exp (−(1.2733 (*t* + 0.0327)^0.4106)	0.9834
	Cur-SLN-FL	*Q* = 95.7775 (1 − exp (−(0.0430 (*t* + 0.6485)^0.8326)	0.9962
Ritger-Peppas	Cur	*Q* = 34.6381 (*t*^0.1329)	0.9011
	Cur-SLN-FL	*Q* = 13.1090 (*t*^0.4668)	0.9833

## Data Availability

The data used to support the findings of this study are included within the article.
